# Condition for Global Stability for a SEIR Model Incorporating Exogenous Reinfection and Primary Infection Mechanisms

**DOI:** 10.1155/2020/9435819

**Published:** 2020-11-17

**Authors:** Isaac Mwangi Wangari

**Affiliations:** Department of Mathematics and Actuarial Science, The Catholic University of Eastern Africa (CUEA), I Langata Main Campus I Bogani East Rd, Off Magadi Rd, P.O. Box 62157-00200 Nairobi, Kenya

## Abstract

A mathematical model incorporating exogenous reinfection and primary progression infection processes is proposed. Global stability is examined using the geometric approach which involves the generalization of Poincare-Bendixson criterion for systems of *n*-ordinary differential equations. Analytical results show that for a Susceptible-Exposed-Infective-Recovered (SEIR) model incorporating exogenous reinfection and primary progression infection mechanisms, an additional condition is required to fulfill the Bendixson criterion for global stability. That is, the model is globally asymptotically stable whenever a parameter accounting for exogenous reinfection is less than the ratio of background mortality to effective contact rate. Numerical simulations are also presented to support theoretical findings.

## 1. Introduction

Mathematical models, in particular, models tracking dynamics of infectious diseases, are of utmost importance due to their application in the assessment of public health policies by national and international agencies. In such models, one of the intriguing aspects that often occurs is when modellers need to know whether the disease will disappear or will permanently remain in the population. This question is answered mainly through investigating the asymptotic stability of the disease-free equilibrium (DFE) as well the endemic equilibrium. It is already known that if the DFE is globally asymptotically stable, then the disease eradication is assured regardless of the initial number of infected individuals in the population [1]. An influx of infected cases may trigger an isolated epidemic outbreak, but they may not make the disease endemic in the population [2]. In contradiction to DFE, if the endemic equilibrium is globally asymptotically stable (GAS) and a few infected individuals are initially introduced, then, the disease will be permanently present in the population.

In the sequel, there are two major methods used in the analysis of global stability of endemic equilibrium: Lyapunov direct method and geometric method. Although the Lyapunov direct method is often used in proving global stability of infectious diseases models, it is sometimes difficult to use because it requires an auxiliary function which is hard to construct. This is because there are no existing general methods for constructing such Lyapunov functions. Moreover, Lyapunov functions for models with parameter(s) that induce bistability phenomena may not even exist. The second method, sometimes referred to as *geometric approach to global stability*, is a generalization of the Poincare-Bendixson criterion for systems of *n* ordinary differential equations. This method was developed by Li and Muldowney [3, 4] in midnineties to address problems encountered with the Lyapunov direct method. The technique is extensively being used to analyze global properties of mathematical models emanating in mathematical epidemiology as well as in other biomathematical contexts. For instance, its applications can be seen in toxicant-population interaction models, Lotka-Volterra models incorporating delay [5, 6], and mathematical epidemic models modelling dynamics of HIV in a human host [7]. Due to mathematical technicalities involved with the geometric approach, it seems to work quite well with low-dimensional mathematical models such as SIR (Susceptible-Infective-Recovered) and SIRS (Susceptible-Infective-Recovered-Susceptible) which can be reduced to bidimensional models (i.e., *n* = 2). Moreover, this method has also been found to be more appropriate in SEIR-like (Susceptible-Exposed-Infective-Recovered) which are represented by a system of four ordinary differential equations (ODEs). This is because their dynamics can be reduced to a three-dimensional system (see [3, 7–11]).

Li and Muldowney [3] proved global stability of a SEIR-like model. However, there are some special cases of SEIR-like models that may not be entirely explained by the global thresholds obtained in [3]. Thus, building on the work of Li and Muldowney, we consider new dynamics that may alter the global stability conditions. For, instance if individuals in incubation period which in this case in compartment *E* experience reinfection, then, new dynamics are likely to arise which may alter the global conditions. Several diseases such as SARS (Severe acute respiratory syndrome), HIV (Human immunodeficiency virus), Ebola, malaria, influenza, and tuberculosis (TB) have an incubation period, and during this stage of infection, individuals can be reinfected by the same or a new strain of the disease (exogenous reinfection).

Castillo-Chavez and Song [12] reviewed the earliest mathematical models of TB dynamics that appeared in the 1960s. Their review investigated several epidemiological factors that are pertinent to TB transmission dynamics. These included the role played by close and casual contacts on TB dynamics, the role of demographic factors (births and deaths), and the role played by intervention strategies implemented to mitigate TB. Further, they extended their review by considering other models such as cell-based models for TB transmission at the immune system level as well as Markov chain models primarily focusing on TB projection. Although these authors considered a SEIT (Susceptible-Exposed-Infective-Treated) model to analyze the local stability of the disease-free equilibrium in the neighbourhood of *R*_0_ = 1, using the famous Castillo-Chavez method derived in [12], they never considered the global properties of the persistent equilibrium. Again, the SEIT proposed model did not incorporate the primary progression pathway in the analysis of the local stability using the Castillo-Chavez method.

It is imperative to note that the Castillo-Chavez et al. [12] method for local stability is used to verify whether a dynamical system exhibits the phenomenon of backward bifurcation. The SEIT model reviewed in [12] obtained a condition for backward bifurcation which is different from the one obtained in the model studied here simply because they omitted the primary progression pathway. The exclusion of primary progression pathway and lack of investigating the global properties of the persistent equilibrium motivated us to attempt to understand the global properties of a SEIR model. Moreover, the model studied here goes beyond understanding the phenomenon of backward bifurcation which is well documented in literature (see [13–18] and the references therein); instead, we attempt to investigate the global properties of a SEIR model incorporating both exogenous reinfection and primary progression infection pathways which was not studied in [12]. The global stability analysis of the persistent equilibrium performed on the proposed SEIR model using the geometric approach is the central feature that distinguishes our model from Castillo-Chavez and Song's [12] paper.

Many infectious diseases in particular those caused by bacterial and viral infections do not render permanent immunity after recovering from the first episode. As a result, they are characterized by partial or complete loss of immunity and subsequent exogenous reinfection. Exogenous reinfection can occur in diseases such as tuberculosis (TB) and flu. Often upon initial infection, individuals pass through different stages before they reach the symptomatic stage where they manifest disease symptoms. Some individuals may pass through a latent stage or dormant state (as in TB or COVID-19) where the disease stays inactive for a specified period of time while some may progress directly to the infectious stage (fast progression or primary progression). An individual infected with TB can either pass through a latent stage or progress directly to the infectious stage (primary progression).

The novelty of this study is the incorporation of exogenous reinfection and primary progression infection mechanisms which were excluded in previous three-dimensional SEIR-like models used to study global stability (see [3, 7, 11, 19]). Thus, our main task is to investigate global properties of a SEIR model including exogenous reinfection and primary progression infection processes using geometric approach. According to our knowledge, the global stability results deduced in this model have not been previously obtained.

## 2. Mathematical Model

The host population is partitioned into four compartments, the susceptible, exposed (latent), infective, and recovered, with subpopulations denoted by *S*, *E*, *I*, and *R*, respectively. The total population at time *t* is represented by *N*(*t*) = *S*(*t*) + *E*(*t*) + *I*(*t*) + *R*(*t*). We assume a frequency-dependent incidence rate (standard incidence rate)

(1) $$\begin{array}{c} \lambda =\frac{c\beta I\left(t\right)}{N\left(t\right)}, \end{array}$$

as the force of infection. Here, *c* represents the host-host contact, *β* is the probability that a contact results in transmission, and *I*(*t*)/*N*(*t*) is the prevalence of infection, sometimes referred to as the “frequency” of infection [20]. After initial infection, a proportion *q* of susceptible individuals can move directly to the infectious stage (primary progression) while the rest move to latent compartment (slow progression), while in latent compartment, individuals are assumed to be exogenously reinfected, hence moving to the infectious stage at a rate *pλE*. Precisely, the subpopulation of susceptibles is generated by recruitment through births and immigration at a rate Λ. The population is decreased due to contact with infectious individuals at a rate *λS*. The exposed subpopulation is generated due to slow progression of the disease at a rate (1 − *q*)*λS*. Moreover, individuals leave the exposed subpopulation due to exogenous reinfection and endogenous reactivation at rates *pλE* and *kE*, respectively. The infected subpopulation is generated by both fast progression and exogenous reinfection at rates *qλE* and *pλE*. It is diminished when individuals recover from disease due to therapy at rate *γI* and disease-related death rate *μ*_*d*_. The recovered subpopulation is generated by recovery of infected individuals at a rate *γ*. All individuals in each subpopulation experience natural death at the same rate through the background mortality rate *μ*. The equation representing transfer of individuals among the compartments is now given by

(2) $$\begin{array}{c} S^{\prime }=\Lambda -\lambda S-\mu S,\\ E^{\prime }=\left(1-q\right)\lambda S-p\lambda E-\left(k+\mu \right)E,\\ I^{\prime }=q\lambda S+p\lambda E+kE-\left(\mu +\gamma +\mu_{d}\right)I,\\ R^{\prime }=\gamma I-\mu R. \end{array}$$

## 3. Existence of the Equilibria

For mathematical tractability, we transform model equation (2) in terms of proportions of the individuals in each compartment. Thus, we define *s* = *S*/*N*, *e* = *E*/*N*, *i* = *I*/*N*, and *r* = *R*/*N* as proportions for the compartments *S*, *E*, *I*, and *R*, respectively. Now differentiating the corresponding proportions with respect to time, it is not difficult to deduce that *s*, *e*, *i*, *r*, and *N* satisfy the following differential equations:

(3) $$\begin{array}{c} s^{\prime }=\frac{\Lambda }{N}-\left[\frac{\Lambda }{N}-\mu_{d}i\right]s-c\beta is,\\ e^{\prime }=\left(1-q\right)c\beta is-pc\beta ie-\left[\frac{\Lambda }{N}-\mu_{d}i\right]e-ke,\\ i^{\prime }=qc\beta is+pc\beta ie+ke-\left[\frac{\Lambda }{N}-\mu_{d}i\right]i-\left(\gamma +\mu_{d}\right)i,\\ r^{\prime }=\gamma i-\left[\frac{\Lambda }{N}-\mu_{d}i\right]r,\\ s+e+i+r=1,\\ N^{\prime }=\left[\frac{\Lambda }{N}-\left(\mu +\mu_{d}i\right)\right]N. \end{array}$$

where *Ω* = {(*s*, *e*, *i*, *r*, *N*) ∈ *ℝ*_+_^5^ : 0 ≤ *s*, 0 ≤ *e*, 0 ≤ *i*, 0 ≤ *r*, *s* + *e* + *i* + *r* ≤ 1, *N* ≤ Λ/*μ*}.

It is easy to observe that the variable *r* in equation (3) does not affect other equations; thus, we can drop the fourth equation. Again, all equations in (3) depend on *N*. So replacing Λ/*N* = *μ* + *μ*_*d*_*i* into the first, second, and third equations, we have the following reduced system:

(4) $$\begin{array}{c} s^{\prime }=\mu +\mu_{d}i-\left(\mu +c\beta i\right)s,\\ e^{\prime }=\left(1-q\right)c\beta is-pc\beta ie-\left(\mu +k\right)e,\\ i^{\prime }=qc\beta is+pc\beta ie+ke-\left(\mu +\gamma +\mu_{d}\right)i. \end{array}$$

It is easy to show that the region *Ω* = {(*s*, *e*, *i*) ∈ *ℝ*_+_^3^ : 0 ≤ *s*, 0 ≤ *e*, 0 ≤ *is* + *e* + *i* ≤ 1}, where the model equation (4) is biologically feasible is positively invariant, where *ℝ*_+_^3^ represents the nonnegative cone of *ℝ*^3^. In the absence of disease, the model equation (4) has an intrinsic equilibrium point *P*_0_ = (1, 0, 0). This equilibrium is the disease-free equilibrium point (DFE).

The basic reproduction number is defined as the number of secondary infections generated by one newly infected individual when introduced into an entirely susceptible population at the disease-free equilibrium point during its mean infective period [1]. The basic reproduction number denoted by *R*_0_ is calculated following the next-generation operator method as developed in Van den Driessche and Watmough [1]. Note that the nonlinear term with new infections *ℱ* and the transition term *𝒱* are, respectively, given by

(5) $$\begin{array}{c} F=\left(\begin{array}{c} \left(1-q\right)c\beta is\\ qc\beta is \end{array}\right),\\ V=\left(\begin{array}{c} \left(\mu +k\right)e\\ \left(\mu +\gamma +\mu_{d}\right)i-ke \end{array}\right). \end{array}$$

The linearized matrices *F* and *V* computed at the disease-free equilibrium *P*_0_ yield

(6) $$\begin{array}{c} F=\left(\begin{array}{cc} 0 & \left(1-q\right)c\beta \\ 0 & qc\beta \end{array}\right),\\ V=\left(\begin{array}{cc} \left(\mu +k\right) & 0\\ -k & \left(\mu +\gamma +\mu_{d}\right) \end{array}\right). \end{array}$$

Hence, the next generation matrix is

(7) $$\begin{array}{c} K=FV^{-1}=\left(\begin{array}{cc} \frac{k\left(1-q\right)c\beta }{\left(\mu +k\right)\left(\mu +\gamma +\mu_{d}\right)} & \frac{\left(1-q\right)c\beta }{\left(\mu +\gamma +\mu_{d}\right)}\\ \frac{kqc\beta }{\left(\mu +k\right)\left(\mu +\gamma +\mu_{d}\right)} & \frac{qc\beta }{\left(\mu +\gamma +\mu_{d}\right)} \end{array}\right). \end{array}$$

One of the eigenvalue of the above matrix is zero while the other (dominant eigenvalue) gives the basic reproduction number. Thus, the basic reproduction number is given as

(8) $$\begin{array}{c} R_{0}=\frac{c\beta \left(k+\mu q\right)}{\left(\mu +k\right)\left(\mu +\gamma +\mu_{d}\right)}. \end{array}$$

It is easy to see that *R*_0_ does not contain parameter *p* which accounts for exogenous reinfection. This indicates that *R*_0_ alone may not sufficiently explain dynamics of model system (4); rather, additional restrictions are needed. Now, we proceed to obtain the nonzero steady states when disease is present in the population. Setting the equations of system (4) to zero and simplifying lead to the following expressions written in terms of *i*^∗^

(9) $$\begin{array}{c} s^{*}=\frac{\mu +\mu_{d}i^{*}}{\mu +c\beta i^{*}},\\ e^{*}=\frac{\left(1-q\right)c\beta i^{*}\left(\mu +\mu_{d}i^{*}\right)}{\left(\mu +c\beta i^{*}\right)\left(pc\beta i+\mu +k\right)}. \end{array}$$

Substituting expression (9) into the third equation of system (4) leads to the following:

(10) $$\begin{array}{c} p\left(i^{*}\right)=i^{*}\left(d_{2}i^{*2}+d_{1}i^{*}+d_{0}\right)=0, \end{array}$$

where

(11) $$\begin{array}{c} d_{2}=\left(\mu +\gamma \right)pc^{2}\beta^{2},\\ d_{1}=\mu pc\beta \left(\mu +\gamma +\mu_{d}\right)+c\beta \left(\mu +\gamma \right)\left(\mu +k\right)+c\beta \mu \mu_{d}\left(1-q\right)-\mu pc^{2}\beta^{2},\\ d_{0}=\mu \left(\mu +k\right)\left(\mu +\gamma +\mu_{d}\right)\left(1-R_{0}\right). \end{array}$$

The root *i*^∗^ = 0 corresponds to a scenario where there is no disease in the population (DFE). The other nonzero roots of model system (4) can be obtained by solving for *i*^∗^ from

(12) $$\begin{array}{c} p_{1}\left(i^{*}\right)=d_{2}i^{*2}+d_{1}i^{*}+d_{0}=0 \end{array}$$

and substituting them in (9).

From equation (12), it is not difficult to see that *d*_2_ is always positive, *d*_0_ > 0⇔*R*_0_ < 1, and *d*_0_ < 0⇔*R*_0_ > 1. Now, by Descartes Rule of Signs, it follows that there is a unique endemic equilibrium whenever *d*_0_ < 0: two positive endemic equilibria if *d*_0_ > 0, *d*_1_ < 0, *d*_1_^2^ − 4*d*_0_*d*_2_ > 0 and no positive endemic equilibria otherwise. Moreover, a bifurcation point occurs when *d*_0_ > 0, *d*_1_ < 0, and *d*_1_^2^ − 4*d*_0_*d*_2_ = 0 (i.e., the point where the two positive endemic equilibria collide, leaving the DFE as the only equilibrium point). At the point where the two positive equilibria (which we shall denote by *R*_0_^*c*^) collide, *R*_0_ = *R*_0_^*c*^. The quantity *R*_0_^*c*^ given in the appendix equation (A.2) can be easily obtained by setting *d*_1_^2^ − 4*d*_0_*d*_2_ = 0 (see the appendix for detailed derivation). Now taking into account the above discussion on equation (12), we deduce Lemma 1.

**Lemma 1 .**

- For *d*_1_ > 0, then, the model equation (4) admits no positive real equilibria whenever *R*_0_ < *R*_0_^*c*^ < 1
- For *d*_1_ < 0, then, the model equation (4) admits two positive endemic equilibria *P*_1_ and *P*_2_ whenever *R*_0_^*c*^ < *R*_0_ < 1
- For *d*_1_ < 0, then, the model equation (4) admits a unique positive endemic equilibrium *P*_∗_ whenever *R*_0_ ≥ 1

The occurrence of two positive endemic equilibria when *R*_0_ < 1 hints the possibility of backward bifurcation phenomenon. Hence, the next section of the work is dedicated on detemining the type of bifurcation exhibited by model equation (4).

## 4. Proof of Existence of Backward Bifurcation

Define

(13) $$\begin{array}{c} p^{c}=\left(\frac{k+\mu q}{\mu \left(1-q\right)}\right)\left(\frac{\mu \mu_{d}\left(1-q\right)+\left(\mu +k\right)\left(\mu +\gamma \right)}{\mu \left(\mu +\gamma +\mu_{d}\right)}\right). \end{array}$$

Then, Theorem 2 follows:

**Theorem 1 .**

- The model equation (4) exhibits backward bifurcation at *R*_0_ = 1 whenever *p* > *p*^*c*^
- The model equation (4) exhibits forward bifurcation at *R*_0_ = 1 whenever *p* < *p*^*c*^

**Proof**

To show that model system (4) exhibits backward bifurcation phenomena, we apply the Center Manifold approach as outlined by Castillo-Chavez and Song in [12]. For clarity and understanding of the center manifold theory, the model equation (4) variables are transformed as follows: *y*_1_ = *s*, *y*_2_ = *e*, *y*_3_ = *i*, and the total population *n* = ∑_*j*=1_^3^*y*_*j*_. Define *Y* = (*y*_1_, *y*_2_, *y*_3_)^*T*^ (*T* denotes transpose), such that the model equation (4) can be rewritten as *dY*/*dt* = *F*(*y*), where *F* = (*f*_1_, *f*_2_, *f*_3_). Hence, it follows

(14) $$\begin{array}{c} y_{1}^{\prime }=\mu +\mu_{d}y_{3}-\mu y_{1}-c\beta y_{1}y_{3}=f_{1},\\ y_{2}^{\prime }=\left(1-q\right)c\beta y_{1}y_{3}-pc\beta y_{2}y_{3}-\left(\mu +k\right)y_{2}=f_{2},\\ y_{3}^{\prime }=qc\beta y_{1}y_{3}+pc\beta y_{2}y_{3}+ky_{2}-\left(\mu +\gamma +\mu_{d}\right)y_{3}=f_{3}. \end{array}$$

Now, let $c\beta =\tilde{\beta }$ and choose $\tilde{\beta }$ as the bifurcation parameter. Note that at *R*_0_ = 1,

(15) $$\begin{array}{c} \tilde{\beta }=\beta^{*}=\frac{\left(\mu +k\right)\left(\mu +\gamma +\mu_{d}\right)}{\left(k+\mu q\right)}. \end{array}$$

Then, the Jacobian matrix of equation (14) evaluated at DFE is given as

(16) $$\begin{array}{c} J_{\left(P_{0}\right)}=\left(\begin{array}{ccc} -\mu & 0 & \mu_{d}-\beta^{*}\\ 0 & -\left(\mu +k\right) & \left(1-q\right)\beta^{*}\\ 0 & k & q\beta^{*}-\left(\mu +\gamma +\mu_{d}\right) \end{array}\right). \end{array}$$

With $\tilde{\beta }=\beta^{*}$, the transformed system (14) has a hyperbolic equilibrium point (i.e., it has a simple eigenvalue with zero real part, and all other eigenvalues are negative). Hence, we can apply the center manifold theory in [12] to analyze dynamics of the transformed system (14) near $\tilde{\beta }=\beta^{*}$. It is easy to obtain the right and left eigenvectors of the Jacobian matrix *J*_(*P*_0_)_, respectively, denoted by *v* = (*v*_1_, *v*_2_, *v*_3_)^*T*^ and *w* = (*w*_1_, *w*_2_, *w*_3_).

(17) $$\begin{array}{c} \text{Right}\text{eigenvectors}:v_{1}=\frac{\mu_{d}-\beta^{*}}{\mu }v_{3},v_{2}=\frac{\left(1-q\right)\beta^{*}}{\mu +k}v_{3},v_{3}=v_{3}>0,\\ \text{Left}\text{eigenvectors}:w_{1}=0,w_{2}=\frac{k}{\mu +k}w_{3}w_{3}=w_{3}>0. \end{array}$$

Now, we proceed to obtain the associated bifurcation parameters, *a* and *b*, as described in Theorem 4.1 of [12], where

(18) $$\begin{array}{c} a=\overset{3}{\underset{k,i,j=1}{\sum }}w_{k}v_{i}v_{j}\frac{\partial^{2}f_{k}\left(0,0\right)}{\partial y_{i}\partial y_{j}},\\ b=\overset{3}{\underset{k,i=1}{\sum }}w_{k}v_{i}\frac{\partial^{2}f_{k}\left(0,0\right)}{\partial y_{i}\partial \beta^{*}}. \end{array}$$

To obtain the associated bifurcation coefficient *a*, we first obtain the nonvanishing partial derivatives of model system (14) evaluated at DFE. Hence, it follows that

(19) $$\begin{array}{c} \frac{\partial^{2}f_{1}\left(0,0\right)}{\partial y_{1}\partial y_{3}}=-\beta^{*},\\ \frac{\partial^{2}f_{2}\left(0,0\right)}{\partial y_{1}\partial y_{3}}=\left(1-q\right)\beta^{*},\\ \frac{\partial^{2}f_{2}\left(0,0\right)}{\partial y_{1}\partial y_{3}}=-p\beta^{*},\\ \frac{\partial^{2}f_{3}\left(0,0\right)}{\partial y_{1}\partial y_{3}}=q\beta^{*},\\ \frac{\partial^{2}f_{3}\left(0,0\right)}{\partial y_{2}\partial y_{3}}=p\beta^{*}, \end{array}$$

so that

(20) $$\begin{array}{c} a=w_{1}v_{1}v_{3}\frac{\partial^{2}f_{1}\left(0,0\right)}{\partial y_{1}\partial y_{3}}+w_{2}v_{1}v_{3}\frac{\partial^{2}f_{2}\left(0,0\right)}{\partial y_{1}\partial y_{3}}+w_{2}v_{2}v_{3}\frac{\partial^{2}f_{2}\left(0,0\right)}{\partial y_{2}\partial y_{3}}+w_{3}v_{1}v_{3}\frac{\partial^{2}f_{3}\left(0,0\right)}{\partial y_{1}\partial y_{3}}+w_{3}v_{2}v_{3}\frac{\partial^{2}f_{3}\left(0,0\right)}{\partial y_{2}\partial y_{3}},=\frac{\mu \left(1-q\right)\beta^{*2}w_{3}v_{3}v_{3}}{{\left(\mu +k\right)}^{2}}\left(p-\left(\frac{k+\mu q}{\mu \left(1-q\right)}\right)\left(\frac{\mu \mu_{d}\left(1-q\right)+\left(\mu +k\right)\left(\mu +r\right)}{\mu \left(\mu +\gamma +\mu_{d}\right)}\right)\right),=\frac{\mu \left(1-q\right)\beta^{*2}w_{3}v_{3}v_{3}}{{\left(\mu +k\right)}^{2}}\left(p-p^{c}\right), \end{array}$$

where

(21) $$\begin{array}{c} p^{c}=\left(\frac{k+\mu q}{\mu \left(1-q\right)}\right)\left(\frac{\mu \mu_{d}\left(1-q\right)+\left(\mu +k\right)\left(\mu +\gamma \right)}{\mu \left(\mu +\gamma +\mu_{d}\right)}\right). \end{array}$$

Moreover, the nonvanishing partial derivatives associated with *b* are

(22) $$\begin{array}{c} \frac{\partial^{2}f_{2}\left(0,0\right)}{\partial y_{3}\partial \beta^{*}}=\left(1-q\right)\beta^{*},\\ \frac{\partial^{2}f_{3}\left(0,0\right)}{\partial y_{3}\partial \beta^{*}}=q\beta^{*}, \end{array}$$

so that

(23) $$\begin{array}{c} b=w_{2}v_{3}\frac{\partial^{2}f_{2}\left(0,0\right)}{\partial y_{3}\partial \beta^{*}}+w_{3}v_{3}\frac{\partial^{2}f_{3}\left(0,0\right)}{\partial y_{3}\partial \beta^{*}}=\frac{\beta^{*}v_{3}w_{3}\left(k+\mu q\right)}{\mu +k}>0. \end{array}$$

The stability of the model system (4) switches at the transcritical point *R*_0_ = 1. According to Theorem 4.1 of [12], it is stated that if both bifurcation coefficients *a* and *b* are positive, then the system exhibits backward bifurcation. Notice that *a* > 0 if and only if *p* > *p*^*c*^ implying that if this condition hold then the model equation (4) will enter into a bistability regime where there is coexistence of two positive endemic equilibria when *R*_0_ < 1, (i.e., backward bifurcation). If *p* < *p*^*c*^, then the model will have forward bifurcation at *R*_0_ = 1.

The type of bifurcation that occurs at *R*_0_ = 1 is primarily determined by exogenous reinfection parameter *p* whenever it exceeds a certain critical value denoted by *p*^*c*^. Thus, the disease can persist even though the reproduction number is less than one. In such case, the disease can only be eliminated if the basic reproduction number is decreased below a certain threshold. That is, *R*_0_ < *R*_0_^*c*^ < 1. Figures 1(a) and 1(b) show the associated forward bifurcation and backward bifurcation, respectively. It is clear that incorporation of exogenous reinfection does induce new dynamics in model system (4) when *R*_0_ < 1.

It is imperative to mention that in the presence of exogenous reinfection, global stability of the endemic equilibrium *P*_∗_ when *R*_0_ > 1 may not be automatically guaranteed. The next section of the work is dedicated on finding under what condition the endemic equilibrium point *P*_∗_ is globally asymptotically stable whenever *R*_0_ > 1.

## 5. Global Stability Using the Poincare-Bendixson Property

Since our objective is to establish global stability of the unique endemic equilibrium *P*_∗_ when *R*_0_ > 1 in the presence of exogenous reinfection parameter *p*, we first briefly outline the general mathematical framework of the procedure as developed in M. Li and J. Muldowney [3, 19].

Suppose the map *y* ↦ *f*(*y*) is a *C*^1^ function for *y* in an open subset *D* ⊂ *ℝ*^*n*^, and consider the following autonomous dynamical system:

(24) $$\begin{array}{c} y^{\prime }=f\left(y\right). \end{array}$$

Let *y*(*t*, *y*_0_) be the solution to equation (24) satisfying *y*(0, *y*_0_) = *y*_0_. Now, we make the following basic assumptions:

(H1) *D* is simply connected.
(H2) There exists a compact absorbing set *K* ⊂ *D*.
(H3) Equation (24) has a unique equilibrium *y*^∗^ in *D*.

Now under the stated assumptions (*H*1)–(*H*3), *y*^∗^ is said to be globally stable in *D* if it is locally stable and all trajectories in *D* converge to the same equilibrium *y*^∗^. That is, system (24) has no nonconstant periodic solutions. It is important to mention that the major role for global stability is determined by the *Bendixson criteria*. For *n* ≥ 2, a *Bendixson criterion* refers to a condition satisfied by field *f* which precludes the existence of nonconstance periodic solutions of equation (24). When *n* = 2 (i.e., the planar case), the classical results (Poincare-Bendixson theorem and Dulac criteria; see [21]) adequately provide such global conditions. For *n* ≥ 3, a remarkable approach for proving global stability can be traced in the work due to Li and Muldowney [3, 4, 19]. In their paper, they showed that if conditions (*H*1)–(*H*3) hold and differential equation (24) fulfills a Bendixson criterion that is robust under *C*^1^ local *ε*− perturbations of *f* at all nonequilibrium nonwandering points for system (24), then *y*^∗^ is globally stable in *D* provided it is stable. Note that a function *g* ∈ *C*^1^(*D* → *ℝ*^*n*^) is called a *C*^1^ local *ε*− perturbation of *f* at *y*_0_ ∈ *D* if there exists an open neighbourhood *U* of *y*_0_ in *D* such that the support sup(*f* − *g*) ⊂ *U* and |*f* − *g*|_*C*^1^_ < *ε*, where |*f* − *g*|_*C*^1^_ = sup{∣*f*(*y*) − *g*(*y*)∣+∣*f*_*y*_(*y*) − *g*_*y*_(*y*)∣:*y* ∈ *D*}. Also, a point *y*_0_ ∈ *D* is said to be nonwandering for system (24) if for any neighbourhood *U* of *y*_0_ in *D* and there exists arbitrary large *t* such that *U*∩*y*(*t*, *U*) ≠ ∅. An example is any equilibrium, alpha limit point, or omega limit point which is nonwandering. We now state the new Bendixson criterion robust under *C*^1^ local *ε*− perturbations and based on the use of the Lozinski measure as developed in [19]. Now, consider the differential equation (24) under the stated assumptions (*H*1)–(*H*3). Let *P*(*y*) be a $n\begin{array}{c} 2 \end{array}\times n\begin{array}{c} 2 \end{array}$ matrix-valued function which is *C*^1^ for *y* ∈ *D*, and consider

(25) $$\begin{array}{c} A=P_{f}P^{-1}+PJ^{\left[2\right]}P^{-1}, \end{array}$$

where *P*_*f*_ is the directional derivative of *P* in the direction of the vector field *f* in system (24) and is defined as

(26) $$\begin{array}{c} {\left(p_{i,j}\left(y\right)\right)}_{f}={\left(\partial p_{i,j}\left(y\right)/\partial x\right)}^{T}.f\left(y\right)=\nabla p_{i,j}.f\left(y\right) \end{array}$$

and *J*^[2]^ represents the second additive compound matrix *J* (that is, *Df*(*y*) = *J*(*y*)). In [22] where relation of compound matrices to differential equations is established, it is shown that for an arbitrary *n* × *n* matrix *J* = *J*_*i*,*j*_, *J*^[2]^ is a $n\begin{array}{c} 2 \end{array}\times n\begin{array}{c} 2 \end{array}$ matrix. For a special case *n* = 3, the second additive compound matrix *J*^[2]^ can be obtained as

(27) $$\begin{array}{c} J^{\left[2\right]}=\left(\begin{array}{ccc} J_{11}+J_{22} & J_{23} & -J_{13}\\ J_{32} & J_{11}+J_{33} & J_{12}\\ -J_{31} & J_{21} & J_{22}+J_{33} \end{array}\right). \end{array}$$

Now consider the following quantity ${\bar{q}}_{2}$ given as

(28) $$\begin{array}{c} {\bar{q}}_{2}=\underset{t\to \infty }{\lim}\sup\underset{y_{0}\in \Omega }{\sup}\frac{1}{t}\int_{0}^{t}\rho \left(A\left(s,y_{0}\right)\right)ds, \end{array}$$

where *ρ*(*A*) is the Lozinski measure of *A* with respect to vector norm ∣·∣ in *ℝ*^*N*^, $N=\left(\begin{array}{c} n\\ 2 \end{array}\right)$, and is defined as

(29) $$\begin{array}{c} \rho \left(A\right)=\underset{h\to 0^{+}}{\lim}\frac{\;|\;1+hA\;|\;-1}{h}, \end{array}$$

(see [23, 24]). In the paper [19], they proved that if conditions (*H*1) and (*H*2) are satisfied, then ${\bar{q}}_{2}<0$, indicating that there are no orbits giving rise to simple closed rectifiable curve in *D* that is invariant for system (24), (that is, periodic orbits, homoclinic orbits, and heteroclinic cycles). Furthermore, it has been remarked in [19] that under the stated assumptions (*H*1)–(*H*3), quantity ${\bar{q}}_{2}<0$ implies the local stability of equilibrium point *y*^∗^. As a result, Theorem 2 is true.

**Theorem 2 (see [19]).**

Assuming that conditions (*H*1)–(*H*3) hold, then, the equilibrium point *y*^∗^ is globally asymptotically stable in *D* if a function *P*(*y*) and a Lozinski measure *ρ* exist such that quantity ${\bar{q}}_{2}<0$.

It is straightforward to see that whenever *R*_0_ > 1, there exist unique and positive endemic equilibria *P*_∗_ (see Lemma 1) for model system (4). The method outlined above requires that (i) the endemic equilibrium *P*_∗_ is unique in the interior of *Ω* (i.e., condition *H*3 holds) and (ii) in the interior of *Ω* there exists an absorbing compact set (condition *H*2 holds). The model equation (4) studied here with the assumption that *R*_0_ > 1 fulfills conditions *H*1–*H*3. It is easy to prove that when *R*_0_ > 1, the disease-free equilibrium *P*_0_ is unstable (see [1]). The instability of the disease-free equilibrium *P*_0_ combined with *P*_0_ ∈ *δΩ* signals uniform persistence [25]. That is, there exists a positive constant *k*_0_ > 0 such that for every solution (*s*(*t*), *e*(*t*), *i*(*t*), *r*(*t*)) of system (4) with (*s*(0), *e*(0), *i*(0), *r*(0)) in the interior of biologically feasible region, *Ω* satisfies

(30) $$\begin{array}{c} \underset{t\to \infty }{\lim}\inf\;|\;s\left(t\right),e\left(t\right),i\left(t\right),r\left(t\right)\;|\;\geq k_{0}. \end{array}$$

Because of boundedness of the region *Ω*, uniform persistence is equivalent to the existence of a compact set in the interior of *Ω* which is absorbing for (4) (see [26]). Hence, condition *H*1 is satisfied. Also, it is shown that whenever *R*_0_ > 1 the model system (4) has only one equilibrium *P*_∗_ in the interior of *Ω*, so that condition *H*3 is verified.

**Theorem 3 .**

Supposing the conditions *R*_0_ > 1 and 0 < *p* < *μ*/*cβ* are satisfied, then the unique endemic equilibrium *P*_∗_ corresponding to the differential equation (4) is globally asymptotically stable with respect to solutions of (4) originating in the interior of *Ω*.

**Proof**

Now, for our model system (4), the task involves showing that quantity ${\bar{q}}_{2}$ is less than zero or establishing condition(s) that may lead to ${\bar{q}}_{2}<0$. In the interior of the biologically feasible region *Ω*, suppose conditions (*H*1)–(*H*3) hold and let *y* = (*s*, *e*, *i*). Let *f*(*y*) be the vector field of system (4). The Jacobian matrix *J* = *∂f*/*∂y* associated with a general solution *y*(*t*) of our system (4) can be obtained as

(31) $$\begin{array}{c} J=\left[\begin{array}{ccc} -\left(\mu +c\beta i\right) & 0 & \mu_{d}-c\beta s\\ \left(1-q\right)c\beta i & -\left(pc\beta i+\mu +k\right) & \left(1-q\right)c\beta s-pc\beta e\\ qc\beta i & pc\beta i+k & qc\beta s+pc\beta e-\left(\mu +\gamma +\mu_{d}\right) \end{array}\right]. \end{array}$$

The second additive compound matrix *J*^[2]^ of *J* is given as

(32) $$\begin{array}{c} J^{\left[2\right]}=\left[\begin{array}{ccc} J_{11} & \left(1-q\right)c\beta s-pc\beta e & -\left(\mu_{d}-c\beta s\right)\\ pc\beta i+k & J_{22} & 0\\ -qc\beta i & \left(1-q\right)c\beta i & J_{33} \end{array}\right], \end{array}$$

where

(33) $$\begin{array}{c} J_{11}=-\left(2\mu +k+c\beta i+pc\beta i\right),\\ J_{22}=qc\beta s+pc\beta e-\left(2\mu +\gamma +\mu_{d}+c\beta i\right),\\ J_{33}=qc\beta s+pc\beta e-\left(2\mu +\gamma +\mu_{d}+k+pc\beta i\right). \end{array}$$

Now based on the model system (4), we choose a suitable vector norm ∣·∣ in *ℝ*^3^ and a 3 × 3 matrix-valued function *P*(*y*). We set *P* as

(34) $$\begin{array}{c} P\left(s,e,i\right)=\left[\begin{array}{ccc} 1 & 0 & 0\\ 0 & \frac{e}{i} & 0\\ 0 & 0 & \frac{e}{i} \end{array}\right]. \end{array}$$

It follows that

(35) $$\begin{array}{c} P_{f}P^{-1}=\mathrm{diag}\left(0,\frac{e^{\prime }}{e}-\frac{i^{\prime }}{i},\frac{e^{\prime }}{e}-\frac{i^{\prime }}{i}\right),\\ PJ^{\left[2\right]}P^{-1}=\left(\begin{array}{ccc} J_{11} & -pc\beta i+\frac{\left(1-q\right)c\beta is}{e} & \left(c\beta s-\mu_{d}\right)\frac{i}{e}\\ \left(k+pc\beta i\right)\frac{e}{i} & J_{22} & 0\\ -qc\beta e & \left(1-q\right)c\beta i & J_{33} \end{array}\right). \end{array}$$

The matrix *A* = *P*_*f*_*P*^−1^ + *PJ*^[2]^*P*^−1^ is thus obtained as

(36) $$\begin{array}{c} A=\left(\begin{array}{ccc} J_{11} & -pc\beta i+\left(1-q\right)c\beta s\frac{i}{e} & \left(c\beta s-\mu_{d}\right)\frac{i}{e}\\ \left(k+pc\beta i\right)\frac{e}{i} & J_{22}+\frac{e^{\prime }}{e}-\frac{i^{\prime }}{i} & 0\\ -qc\beta e & \left(1-q\right)c\beta i & J_{33}+\frac{e^{\prime }}{e}-\frac{i^{\prime }}{i} \end{array}\right). \end{array}$$

Now, matrix *A* can be rewritten in block form as

(37) $$\begin{array}{c} A=\left[\begin{array}{cc} A_{11} & A_{12}\\ A_{21} & A_{22} \end{array}\right], \end{array}$$

where

(38) $$\begin{array}{c} A_{11}=-\left[2\mu +k+c\beta i+pc\beta i\right],\\ A_{12}=\left[-pc\beta i+\left(1-q\right)c\beta s\frac{i}{e},\left(c\beta s-\mu_{d}\right)\frac{i}{e}\right],\\ A_{21}=\left[\begin{array}{c} \left(k+pc\beta i\right)\frac{e}{i}\\ -qc\beta e \end{array}\right],\\ A_{22}=\left[\begin{array}{cc} J_{22}+\frac{e^{\prime }}{e}-\frac{i^{\prime }}{i} & 0\\ \left(1-q\right)c\beta i & J_{33}+\frac{e^{\prime }}{e}-\frac{i^{\prime }}{i} \end{array}\right]. \end{array}$$

Following [19], we let (*u*, *v*, *w*) represent the vectors in ${\mathbb{R}}^{3}≅{\mathbb{R}}^{3\begin{array}{c} 2 \end{array}}$. Now, for the norm |·| in *ℝ*^3^, select

(39) $$\begin{array}{c} \left|u,v,w\right|=\max\left\{\left|u\right|,\left|v\right|+\left|w\right|\right\}, \end{array}$$

and let *ρ* represent the Lozinskii measure with respect to this norm. Applying the method of approximating the *ρ*(*A*) as given in [24], we have

(40) $$\begin{array}{c} \rho \left(A\right)\leq \sup\left\{g_{1},g_{2}\right\}, \end{array}$$

where

(41) $$\begin{array}{c} g_{1}=\rho_{1}\left(A_{11}\right)+\left|A_{12}\right|,\\ g_{2}=\left|A_{21}\right|+\rho_{1}\left(A_{22}\right). \end{array}$$

Note that in equation (41), |*A*_12_| and |*A*_21_| are operator norms of *A*_12_ and *A*_21_ with respect to the *l*_1_ vector norm when they are regarded as mapping from *ℝ*^2^ to *ℝ* and *ℝ*^2^ to *ℝ*, respectively. *ρ*_1_(*A*_22_) represents the Lozinskii measure of the 2 × 2 matrix *A*_22_ with respect to the *l*_1_ norm in *ℝ*^2^. To obtain *ρ*_1_(*A*_22_), we sum the absolute value of the off-diagonal elements to the diagonal one in each column of *A*_22_ and then take the maximum of two sums. Now, it follows that

(42) $$\begin{array}{c} \rho_{1}\left(A_{11}\right)=-\left(2\mu +k+c\beta i+pc\beta i\right),\\ \rho_{1}\left(A_{22}\right)=qc\beta s+pc\beta e+\left(1-q\right)c\beta i+\frac{e^{\prime }}{e}-\frac{i^{\prime }}{i}-\left(2\mu +\gamma +\mu_{d}+c\beta i\right),\\ \;|\;A_{12}\;|\;=\max\left[\frac{c\beta si}{e}-\frac{qc\beta si}{e}-pc\beta i,\frac{c\beta si}{e}-\frac{\mu_{d}i}{e}\right]=\frac{c\beta si}{e}-\min\left\{pc\beta i+\frac{qc\beta si}{e},\frac{\mu_{d}i}{e}\right\},\\ \;|\;A_{21}\;|\;=\max{\left[\left(k+pc\beta i\right)\frac{e}{i},-qc\beta e\right]}^{T}=\left(k+pc\beta i\right)\frac{e}{i}. \end{array}$$

Now we have

(43) $$\begin{array}{c} g_{1}=\frac{c\beta si}{e}-\left(2\mu +k+c\beta i+pc\beta i\right)-\min\left\{pc\beta i+\frac{qc\beta si}{e},\frac{\mu_{d}i}{e}\right\},\\ g_{2}=\left(k+2pc\beta i\right)\frac{e}{i}+qc\beta s+\frac{e^{\prime }}{e}-\frac{i^{\prime }}{i}-qc\beta i-\left(2\mu +\gamma +\mu_{d}\right). \end{array}$$

Note that in system (4), second and third equations can, respectively, be written as

(44) $$\begin{array}{c} \frac{e^{\prime }}{e}-\frac{c\beta is}{e}+\frac{qc\beta is}{e}=-\left(pc\beta i+\mu +k\right),\\ \frac{i^{\prime }}{i}+\left(\mu +\gamma +\mu_{d}\right)=pc\beta e+qc\beta s+\frac{ke}{i}. \end{array}$$

Now substituting equality (44) into equation (43) and equality (44) into equation (43) leads to

(45) $$\begin{array}{c} g_{1}=\frac{e^{\prime }}{e}-\mu -c\beta i-\min\left\{pc\beta i,\frac{\mu_{d}i}{e}\right\}\\ \leq \frac{e^{\prime }}{e}-\mu ,\\ g_{2}=\frac{e^{\prime }}{e}-\mu -qc\beta i+pc\beta e,\\ \leq \frac{e^{\prime }}{e}-\mu +pc\beta e,\\ \leq \frac{e^{\prime }}{e}-\mu +pc\beta \left(\text{because}0<\text{s},\text{e},\text{i}\leq 1\right). \end{array}$$

Thus, we have

(46) $$\begin{array}{c} \rho \left(A\right)\leq \sup\left(g_{1},g_{2}\right)\leq \sup\left\{\frac{e^{\prime }}{e}-\mu ,\frac{e^{\prime }}{e}-\mu +pc\beta \right\}\leq \frac{e^{\prime }}{e}-\mu +pc\beta . \end{array}$$

Hence, we now have

(47) $$\begin{array}{c} \rho \left(A\right)\leq \frac{e^{\prime }}{e}-\mu +pc\beta . \end{array}$$

Integrating both sides of equation (47) at the same time for $t>\bar{t}$, we get

(48) $$\begin{array}{c} {\bar{q}}_{2}=\frac{1}{t}\int_{0}^{t}\rho \left(A\right)ds=\frac{1}{t}\int_{0}^{\bar{t}}\rho \left(A\right)ds+\frac{1}{t}\int_{\bar{t}}^{t}\rho \left(A\right)ds,\\ \leq \frac{1}{t}\log\frac{e\left(t\right)}{e\left(\bar{t}\right)}+\frac{1}{t}\int_{0}^{\bar{t}}\rho \left(A\right)ds-\left(\mu -pc\beta \right),\\ \Rightarrow {\bar{q}}_{2}=\underset{t\to \infty }{\lim}\text{supsup}\frac{1}{t}\int_{0}^{t}\rho \left(A\right)ds<-\left(\mu -pc\beta \right)<0. \end{array}$$

and the Bendixson criterion given by equation (28) is verified. Observe that ${\bar{q}}_{2}<0$ under condition that 0 < *p* < *μ*/*cβ*. Thus, the proof of Thoerem (3) is complete.

## 6. Numerical Analysis

Numerically, it is possible to verify the validity of Theorem 4. Recalling that for model equation (4) to be globally stable, the condition 0 < *p* < *μ*/*cβ* must be fulfilled. Now, we numerically investigate two scenarios numerically: that is, where condition *p* < *μ*/*cβ* and where *p* > *μ*/*cβ*.

- By choosing the following set of hypothetical parameters, *μ* = 0.017, *μ*_*d*_ = 0.1, *k* = 0.001, *γ* = 2, *q* = 0.05, *p* = 0.0005, *c* = 60, *β* = 0.519 and initial conditions *s* = 1, *e* = 0, *i* = 0.00001, with these parameter values, condition *p* < *μ*/*cβ* is satisfied. That is, *p* = 0.0005 < *μ*/*cβ* = 0.00055. Figure 2 shows that model system (4) is globally asymptotically stable whenever condition *p* < *μ*/*cβ* is satisfied. That is, there are no periodic solutions
- Now, we choose another set of parameter values that satisfy the condition *p* > *μ*/*cβ*, namely, *μ* = 0.017, *μ*_*d*_ = 0.1, *k* = 0.001, *γ* = 2, *q* = 0.05, *p* = 0.135, *c* = 60, *β* = 0.519, and *k*_0_ = 0.019. The initial conditions used are the same as in Case (i) above.  Figure 3 depicts that model system (4) has sustained periodic solutions if condition *p* > *μ*/*cβ*

## 7. Conclusion

A mathematical model is proposed, and its global stability property is analyzed using the geometric approach. The model incorporated exogenous reinfection and primary progression infection processes which were excluded in previous SEIR-like models used to investigate global stability through the Bendixson criterion. The analysis of endemic equilibrium points reveals that the model exhibits backward bifurcation phenomena where two positive endemic equilibria coexist when basic reproduction number is below one.

To investigate global stability, we applied geometric approach and found that the Bendixson criterion cannot be satisfied unless the exogenous reinfection parameter *p* is less than the ratio of background mortality rate (*μ*) to effective contact rate (*cβ*). Interestingly, the primary progression parameter *q* does not impact the condition for global stability for a disease model that follows Susceptible-Exposed-Infective-Recovered stages. Numerically, we verified the validity of global asymptotic stability condition in Theorem 4 and found that it does act as the stability condition for the proposed SEIR model with exogenous reinfection and primary progression infection processes.

## Figures and Tables

**Figure 1:** Illustration of type of bifurcation. (a) Represents forward bifurcation. Parameters used include *μ* = 0.016, *μ*_*d*_ = 0.1, *k* = 0.001, *γ* = 2, *q* = 0.05, *c* = 45, *β* ∈ {0.42,0.45}, and *p* = 0.1245 < *p*^*c*^ = 0.1252. (b) Represents backward bifurcation. Parameters used are the same as in (a) except *p* = 0.15 > *p*^*c*^ = 0.1252. *β*^∗^ = 0.444 corresponds to *R*_0_ = 1. In both figures, the red solid line represents unstable equilibria while the blue solid line represents stable equilibria.

**Figure 2:** Illustration of nonexistence of periodic solutions when condition *p* < *μ*/*cβ* holds true. The corresponding *R*_0_ with the given parameter values is *R*_0_ = 1.5118 > 1.

**Figure 3:** Illustration of existence of periodic solutions when *p* > *μ*/*cβ*. The corresponding *R*_0_ with the given parameter values is *R*_0_ = 1.5118 > 1.

## Data Availability

The current research does not contain any data.

## Appendix

### A. Computation of *R*_0_^*c*^

For simplification, we first rewrite equation (12) coefficients as *d*_1_ = *β*(*b*_1_ − *b*_2_*β*), *d*_0_ = *c*_1_ − *c*_2_*β*, and *d*_2_ = *dβ*^2^, where

(A.1) $$\begin{array}{c} b_{1}=\mu pc\left(\mu +\gamma +\mu_{d}\right)+c\left(\mu +\gamma \right)\left(\mu +k\right)+c\mu \mu_{d}\left(1-q\right),\\ b_{2}=\mu pc^{2},\\ c_{1}=\mu \left(\mu +k\right)\left(\mu +\gamma +\mu_{d}\right),\\ c_{2}=\mu c\left(k+\mu q\right),\\ d=\left(\mu +\gamma \right)pc^{2}. \end{array}$$

Then, choosing *β* as the bifurcation parameter and setting Δ = *d*_1_^2^ − 4*d*_0_*d*_2_ = 0, we obtain the following equation in terms of *β*:

(A.2) $$\begin{array}{c} \Delta \left(\beta \right)=b_{2}^{2}\beta^{2}+2\beta \left(2dc_{2}-b_{1}b_{2}\right)+b_{1}^{2}-4c_{1}d=0. \end{array}$$

Solving equation (A.2), we obtain

(A.3) $$\begin{array}{c} \beta^{c}=\frac{\left(b_{1}b_{2}-2dc_{2}\right)+2\sqrt{d^{2}c_{2}^{2}+db_{2}\left(c_{1}b_{2}-c_{2}b_{1}\right)}}{b_{2}^{2}}>0. \end{array}$$

Finally, replacing *β* with *β*^*c*^ in *R*_0_ (see equation (8)), we obtain

(A.4) $$\begin{array}{c} R_{0}^{c}=\frac{c\beta^{c}\left(k+\mu q\right)}{\left(\mu +k\right)\left(\mu +\gamma +\mu_{d}\right)}. \end{array}$$
